# Deconstruction of the Prevention of Knee Osteoarthritis by Swimming Based on Data Mining Technology

**DOI:** 10.1155/2022/1001686

**Published:** 2022-08-16

**Authors:** Jianxia Yin, Qing Li, Yao Song

**Affiliations:** ^1^Swimming Teaching and Research Office, Xi'an Physical Education University, Xi'an, 710068 Shaanxi, China; ^2^Competition Training Division, Xi'an Physical Education University, Xi'an, 710068 Shaanxi, China

## Abstract

With the continuous development of big data and the continuous improvement of people's living standards, increasingly attention is paid to physical health. Swimming in this sport is effective in preventing the occurrence of arthritis. This paper analyzes the prevention and exploration of arthritis and relies on the traditional method of retrieving clinical literature on the treatment of knee osteoarthritis with traditional Chinese medicine and internal medicine, which requires a lot of manpower and material resources. At this time, the role of data mining technology is brought into play. This article analyzes the prevention of arthritis by swimming. If you rely on the traditional retrieval of clinical literature on the treatment of knee osteoarthritis with traditional Chinese medicine and internal medicine, you will find a lot of disordered data. It takes a lot of manpower and material resources to sort out the summary, and at this time, the role of data mining (DM) technology is brought into play. In this paper, the relevant information of the literature that meets the requirements is established in an Excel database, and the data of the relevant information is entered. Through sorting and analysis, the TCM syndrome types of knee osteoarthritis are summarized. Then, DM technology was used to carry out statistical analysis of frequency and prescription, to summarize the distribution characteristics of the corresponding knee osteoarthritis, TCM syndrome types, and the weight of each syndrome type, and to make a preliminary discussion at the same time. Finally, it is concluded that there are better prevention methods for arthritis in the research methods of traditional Chinese medicine. DM technology has been increasingly applied to all aspects of traditional Chinese medicine. DM technology has improved its research efficiency by 38% and achieved great results, which will play a greater role in promoting the research process of TCM syndrome.

## 1. Introduction

In today's era of rapid development of knowledge economy, with the rapid development of information industrialization and database technology, all walks of life are facing a rapid increase in the amount of data in the process of production practice. There is often a lot of important and useful information hidden behind the surge of data. People urgently need to apply the technology of “removing the rough and saving the fine” and “removing the false and saving the truth” to conduct a systematic and comprehensive analysis and to analyze these higher-level and comprehensive data. From this, DM technology is produced accordingly. The big data platform is built on the distributed storage system and distributed computing system. The distributed system is composed of some inexpensive and cost-effective machines, and dynamic expansion can be achieved by dynamically adding clusters. The dynamic expansion of the cluster can be realized by dynamically adding cheap PCs in the cluster, and the data storage capacity and processing efficiency can be improved, thereby saving resources. Therefore, the use of DM technology to comprehensively analyze, convert it into useful knowledge, explore the laws contained therein, and accelerate the utilization and dissemination of TCM informatization has become the key to the innovation and development of TCM.

Swimming has a preventive effect on arthritis, and a small proportion of patients fail to achieve satisfactory clinical outcomes after knee arthroplasty, which may suggest that existing postoperative rehabilitation models may not be the most effective. Vadher et al. conducted the Post-Knee Replacement Community Rehabilitation Trial, which then evaluated the effects of a new community-based rehabilitation program after knee replacement compared with usual care [1]. Wang et al. have conducted several clinical studies to evaluate the effect of neuromuscular exercise therapy on joint stability in patients with knee osteoarthritis [2]. Li et al., who aimed to systematically evaluate the effect of motor imagery on improvement in functional performance in patients with total knee arthroplasty, included randomized controlled trials evaluating the effect of motor imagery on motor imagery [3]. These articles have well explained the importance of protecting the knee, but they have not been studied on the basis of swimming movement under DM and have certain limitations.

DM technology is a process of extracting some relatively secret but potentially useful information from a large amount of data. Wang et al. excavated the relevant knowledge of extraction parameters from the historical data of the extraction process of traditional Chinese medicine and used it to guide the technicians to select the influencing factors of the orthogonal test and the level of each factor [4]. Using the theoretical basis of 5G and association analysis data mining, Li et al. designed a data model of tennis technical offensive tactics and association rules, which can calculate the distribution rate of certain methods [5]. Many heuristics have been proposed before to build near-optimal decision trees. However, most of them have the disadvantage that only local optima can be obtained. To solve the above problems, Wang et al. proposed a new algorithm with a new segmentation criterion and a new decision tree construction method [6]. Andrew recorded weather events and the resulting road surface conditions during preprocessing and during subsequent events using visual assessments and limited road grip tester assessments. In addition, he conducted extensive laboratory research to complement fieldwork. The combined findings form a decision tree to aid in operational planning and preprocessing [7]. Baneshi et al. proposed a tree-based model to assess the impact of different religious dimensions based on risk factors [8]. Although the above scholars have achieved some practical results, there are still some targeted researches; so, it is necessary to further improve.

In this paper, DM technology is used to analyze the clinical literature of knee osteoarthritis. Through bold innovation and exploration, common single and compound syndrome types in clinical practice were obtained in this study, but it is still dominated by compound syndrome types. Most of the syndrome types of this disease have the compound syndrome type of liver and kidney deficiency syndrome, which will provide a theoretical basis for syndrome differentiation and treatment, and improve the clinical efficacy of knee osteoarthritis. The novelty of the article is as follows: this article will try to analyze and study the clinical syndromes of knee osteoarthritis by relying on the existing clinical literature without the support of clinical research and strive to explore the practical value of the literature so that it can be more reasonably applied in clinical practice.

## 2. DM Technology

### 2.1. Similarity Calculation Method in KNN Algorithm

The KNN algorithm uses a similarity calculation method, arranges and combines according to the degree of similarity, extracts the first *K* objects, uses the similarity between the first *K* objects and the target object as the weight, and then weights the sum. Finally, the result is normalized by the sum of the similarity between the top *K* objects and the target object [9].

#### 2.1.1. Euclidean Distance Method

(1) $$\begin{array}{c} M\left(m_{a},m_{b}\right)=\sqrt{\frac{1}{X}\left(\sum {\left(n_{ak}-n_{bk}\right)}^{2}\right)}. \end{array}$$

In the formula, it is assumed that the feature vector of one text is *m*_*a*_, the feature vector of another text is *m*_*b*_, *X* is the dimension of the feature vector, and *n*_*k*_ represents the *k*-th dimension, because it treats the differences between different properties of the samples as equals, which sometimes does not meet the actual requirements, and does not take into account the influence of the overall variation on the distance.

#### 2.1.2. Angle Cosine Method

(2) $$\begin{array}{c} \text{Sim}\left(m_{a},m_{b}\right)=\frac{\sum n_{ak}\times n_{bk}}{\sqrt{\left(\sum {n^{2}}_{ak}\right)\left(\sum {n^{2}}_{bk}\right)}}. \end{array}$$

The meaning of each parameter is consistent with the Euclidean distance method.

#### 2.1.3. Weight Calculation Formula

(3) $$\begin{array}{c} q\left(y,v_{a}\right)=\sum \text{S}\text{im}\left(y,m_{b}\right)q\left(m_{a},v_{a}\right). \end{array}$$

The *K* training texts calculate the weight of each category in turn, and then the test texts are divided into the categories with the largest weight. Among them, Sim(*y*, *m*_*b*_) is the similarity between the text to be classified and the training text, and *q*(*m*_*b*_, *v*_*a*_) is the category attribute function, when the text *m*_*a*_belongs to category *v*_*a*_, *q*(*m*_*a*_, *v*_*a*_) = 1; otherwise, *q*(*m*_*a*_, *v*_*a*_) = 0.

The traditional KNN algorithm still has many shortcomings when dealing with big data. The first is that all training samples need to be stored, and the second is that the amount of calculation is large; so ,errors are prone to occur in the calculation process. Here, an improved KNN algorithm based on clustering, denoising, and density clipping is proposed.

#### 2.1.4. Application of Density Cropping Based on Clustering Denoising in KNN Algorithm

The traditional KNN algorithm still has many shortcomings when dealing with big data. Here, an improved KNN algorithm based on clustering, denoising, and density clipping is proposed.

As can be seen from Figure 1, even for samples of the same category, due to the differences between samples, and each sample has different representation capabilities for the category, there is a large difference in the degree of similarity between samples.

### 2.2. Naive Bayes

(4) $$\begin{array}{c} P\left(Y\left|X\right.\right)=\frac{P\left(Y\right)P\left(X\left|Y\right.\right)}{P\left(X\right)}. \end{array}$$

*P*(*Y*|*X*) refers to the probability that event *Y* occurs under the condition that event *X* occurs, *P*(*Y*|*X*) refers to the probability that event *X* occurs under the condition that event *Y* occurs, and *P* (*X*) and *P* (*Y*) represent the probability of event *X* and event *Y*, respectively, where event *X* and event *Y* are two independent events [10].

Assuming that there are *m* classified samples in the training sample *M*, the sample attribute *N* = {*n*_1_, *n*_2_ ⋯ *n*_*k*_} belongs to the *c* class, and *n*_*i*_ represents the *i*-th attribute in the sample. According to Bayes' theorem, there are

(5) $$\begin{array}{c} P\left(c\left|\text{N}\right.\right)=\frac{P\left(N\left|\text{c}\right.\right)P\left(c\right)}{P\left(N\right)}. \end{array}$$

For the unknown sample *N*, calculate the conditional probability that the sample is each class, and the class corresponding to the maximum probability value is determined as the class to which the sample belongs. Using the property independence assumption, *P*(*N*|*c*) can be transformed into

(6) $$\begin{array}{c} P\left(N\left|c\right.\right)=\overset{k}{\underset{i=1}{\prod }}P\left(n_{i}\left|c\right.\right). \end{array}$$

Therefore, the Bayesian classification algorithm expression can be written as

(7) $$\begin{array}{c} h\left(N\right)=\arg\max P\left(c\right)\overset{k}{\underset{i=1}{\prod }}P\left(n_{i}\left|c\right.\right). \end{array}$$

### 2.3. Logistic Regression

The regression coefficient is a parameter that represents the influence of the independent variable *x* on the dependent variable *y* in the regression equation. The larger the regression coefficient, the greater the influence of *x* on *y*. As the core algorithm of logistic regression [11], the sigmoid function is calculated as follows:

(8) $$\begin{array}{c} d=\frac{1}{1-e^{-x}}. \end{array}$$

Figure 2 is a graph of the sigmoid function, which converts the *x* value to a *d* value of 0 or 1. Among them, *x* is a regression function, set the regression coefficient *δ*, the input is *M*, and then *x* = *δ*^*T*^*M* and bring it into the above formula to get

(9) $$\begin{array}{c} d=\frac{1}{1-e^{-\left(\delta^{T}M\right)}}. \end{array}$$

It can be transformed into

(10) $$\begin{array}{c} \ln\frac{d}{1-d}=\delta^{T}M. \end{array}$$

If *d* is the probability of a sample *M*, 1-*d* is the inverse probability of *M*, and ln(1/1 − *d*) is the relative probability of *M*.

### 2.4. Support Vector Machines

Support vector machines can be used not only for classification tasks but also for regression tasks. For binary classification problems, it is necessary to draw a hyperplane between different classes to separate the two classes [12]. The equation description of the hyperplane is

(11) $$\begin{array}{c} \omega^{T}x+a=0. \end{array}$$

*ω* = (*ω*_1_, *ω*_2_ ⋯ *ω*_*k*_) is the normal vector of the hyperplane, representing the direction of the plane, and *a* is the displacement, representing the distance between the hyperplane and the origin. In this way, the distance from the point in the sample to the hyperplane is

(12) $$\begin{array}{c} r=\frac{\left|\omega^{T}x+a\right|}{\left\|\omega \right\|}. \end{array}$$

If the hyperplane can separate positive and negative samples, then

(13) $$\begin{array}{c} \left\{\begin{array}{c} \omega^{T}x_{i}+a\geq 1,y_{i}=+1,\\ \omega^{T}x_{i}+a\leq 1,y_{i}=-1. \end{array}\right. \end{array}$$

The sum of the distances from two support vectors of different types to the hyperplane is

(14) $$\begin{array}{c} R=\frac{2}{\left\|\omega \right\|}. \end{array}$$

Moreover, known as “interval,” to find the hyperplane that can maximize the interval, that is, to maximize *R* under the condition of satisfying Equation (13), that is,

(15) $$\begin{array}{c} \begin{array}{c} \underset{\omega ,a}{\max}\frac{2}{\left\|\omega \right\|}\\ s.t.y_{i}\left(\omega^{T}x_{i}+a\right)\geq 1,i=1,2\cdots k \end{array}. \end{array}$$

Maximizing 1/‖*ω*‖ is equivalent to minimizing ‖*ω*‖^2^, and the above formula can be changed to

(16) $$\begin{array}{c} \begin{array}{c} \underset{\omega ,k}{\min\frac{1}{2}{\left\|\omega \right\|}^{2}}\\ s.t.y_{i}\left(\omega^{T}x_{i}+a\right)\geq 1,i=1,2\cdots k \end{array}. \end{array}$$

### 2.5. Decision Tree

The decision tree algorithm is an instance-based inductive learning method. It is a modeling method that uses the tree structure from root to branch to branch. ID3 is a classification algorithm for decision tree learning. The ID3 algorithm is mainly divided according to the size of the information gain and then constructs a decision tree, which is suitable for discrete data. Which attribute is selected in each node in the decision tree is the core of the ID3 algorithm. Its task is to minimize the number of nodes on the decision tree. The smaller the number of nodes, the higher the recognition rate [13].

Assuming that the training set is *M*, the proportion of the *k*-th sample is *P*_*k*_, and the discrete attribute *b* has *V* values of *b*_1_, *b*_2_ ⋯ *b*_*V*_, among which the sample with the attribute value of *b*_*V*_ in the training set is called *M*_*V*_. The first is the concept of information entropy. Information entropy is an indicator to measure the purity of the sample set, which is defined as

(17) $$\begin{array}{c} \text{Ent}\left(M\right)=-\overset{k}{\underset{i=1}{\sum }}p_{i}\log_{2}p_{k}. \end{array}$$

The smaller the information entropy, the higher the purity. The information gain is the gain obtained when the calculation attribute *b* divides the sample *M*, expressed as

(18) $$\begin{array}{c} \text{Gain}\left(M,b\right)=-\overset{k}{\underset{i=1}{\sum }}\frac{\left|M_{V}\right|}{\left|M\right|}\text{Ent}\left(M_{V}\right). \end{array}$$

The gain rate is defined as

(19) $$\begin{array}{c} \text{Gain}\_\text{ratio}\left(M,b\right)=\frac{\text{Gain}\left(D,b\right)}{IV\left(b\right)}. \end{array}$$

Among them,

(20) $$\begin{array}{c} \text{IV}\left(b\right)=-\overset{V}{\underset{V=1}{\sum }}\frac{\left|M_{V}\right|}{\left|M\right|}\log_{2}\frac{\left|M_{V}\right|}{\left|M\right|}. \end{array}$$

This is a fixed value. The characteristic of this value is that the more possible the values of the attribute, the larger the value, which effectively avoids the possibility that the attribute with more values will be preferentially selected.

## 3. Deconstruction of the Effect of Swimming on Knee Osteoarthritis Based on DM Technology

### 3.1. Overview

Knee osteoarthritis is a relatively common chronic joint disease, which is characterized by changes in noninflammatory articular cartilage and bone hyperplasia at the joint edge. Arthritis is more common in middle-aged and elderly patients, and the prevalence of women is twice as high as that of men. The main clinical manifestations are knee joint swelling and pain, morning stiffness, interlocking feeling, and poor mobility. In the later stage, it may progress to muscle atrophy, even varus deformity of the knee joint, and eventually develop the disability of the patient's limbs [14]. The development process of the disease is hidden, which greatly harms people's health and becomes the first cause of sports and chronic disability in the middle-aged and elderly.

Traditional Chinese medicine has many methods for the treatment of knee osteoarthritis, with few side effects and low medical expenses; so, it has the advantage of being extensive and suitable for different types of people and syndrome types in different periods. However, the current research results on the standardization of TCM syndromes for knee osteoarthritis show that there is still no objective and unified standard for syndrome differentiation. It is because the current diagnostic criteria for existing syndrome types are mainly derived from collective research and discussion by some experts. They may not fully agree on the etiology and pathogenesis of knee osteoarthritis, and there are still many different opinions and differences on the syndrome differentiation of the disease: they stay on the personal experience reports or mainly from the statistical results of questionnaires in some areas or special prescriptions based on disease differentiation, resulting in extremely confusing clinical syndrome classification. This makes the implementation and promotion of many effective treatment methods impossible, and the progress of traditional Chinese medicine in the treatment of knee osteoarthritis is also greatly limited [15].

It can be seen that it is essential to standardize the TCM syndrome types of knee osteoarthritis, which will provide a strong theoretical basis for the treatment of knee osteoarthritis based on syndrome differentiation. This helps guide clinical medication and active prevention, which has an important and far-reaching impact on relieving patients' suffering, improving personal quality of life, which helps to guide clinical medication and active prevention, and which is important for alleviating the pain of patients, improving the quality of personal life, and promoting social harmony.

### 3.2. Prevention of Arthritis by Swimming

When patients with knee osteoarthritis swim in water, they will find that the force of water can have a better and obvious therapeutic effect on the joints and relax the joints. At the same time, people reduce the pressure on the joints when swimming; so, the muscles are fully trained, which relieves inflammation and promotes the recovery of various functions to a certain extent. And because synovial fluid is the nutrition of articular cartilage, during exercise, the cartilage accelerates the circulation of synovial fluid during the occasional stress process, so that the condition of arthritis can be relieved.

The horizontal spine of the body during swimming significantly reduces the burden on the spine, relieves the manifestations of pain and inflammation, and has the effect of physical therapy. Dorsiflexing the head from time to time during freestyle and breaststroke stretches the spine of people who work with their heads down for long periods of time. For the elderly, moderate swimming can also prevent osteoporosis, reduce the risk of fractures, improve the function of multiple organs such as the heart and lungs, and improve their own immunity.

### 3.3. Resolve Methods

1. This article determines the clinical literature that needs to be studied according to the research scope, inclusion criteria, and exclusion criteria
2. In the valid clinical literature, general information such as literature titles, authors, research objects, syndrome type, prescription names, treatment principles, prescription, and other related information are summarized and entered into Excel sheet in turn to establish a relevant information database
3. There is data preprocessing for some TCM syndrome types that are not clearly proposed in the effective clinical literature on knee osteoarthritis. However, the treatment principles of prescription are clearly stated, and the types of TCM syndromes are deduced through the reverse syndrome differentiation process of “testing syndromes by method”. To test by method is actually to extract some parts from a certain model and then give the corresponding prescription. After checking the indicators, compare the differences between before and after and between each group according to a certain method. At the same time, the TCM syndrome types are merged and standardized, and finally, a unified and standardized TCM syndrome type is formed
4. It uses the software to perform statistical analysis on the general data (average age, gender) and TCM syndrome types of research objects in the database using DM technology. And the frequency statistical analysis method is used to summarize the average age and gender of the research subjects in the incidence of knee osteoarthritis and the percentage of common clinical TCM syndrome types in the total number of cases and make corresponding charts
5. According to the statistical results of the above data, it is possible to understand the average age and gender of patients in the incidence of knee osteoarthritis, the distribution of common clinical syndrome types, and the weight of each syndrome type. There is a preliminary discussion to establish a more normative, objective, and standard clinical syndrome classification system. The specific process is shown in Figure 3

### 3.4. Deconstruction

#### 3.4.1. Age

The mean age of subjects with knee osteoarthritis was adjusted according to the new regulations in a database of 1270 valid articles. At the same time, mining and analyzing these data, according to the following table, it can be concluded that middle-aged and elderly people over 45 years old are the high-risk group of knee osteoarthritis.  Table 1 is for details about the distribution of relevant information.

#### 3.4.2. Gender

From a database of 1270 valid literatures, 120 patients were extracted for analysis. Among them, there were 20 male patients and 100 female patients, with a male-to-female ratio of 1 : 5. It can be seen that females account for a larger proportion of arthritis cases.

#### 3.4.3. Frequency of Certificate Types

First, standardize the names of 36 related clinical syndrome types by statistical analysis [16]. Statistical analysis will then summarize the relevant 36 types of clinical syndrome names for merging, such as insufficiency of kidney yin or deficiency of kidney yang or deficiency of yin and fire or deficiency of the liver and kidney or deficiency of kidney yuan or deficiency of both yin and yang of the kidney is combined as a syndrome of deficiency of the liver and kidney; wind-cold dampness soaking or cold-damp obstruction or rheumatic obstruction combined with wind-cold-damp obstruction syndrome; collateral obstruction or blood stasis blocking collaterals or meridian blockage or unfavorable meridian combined into tendon and meridian stasis syndrome; damp-heat soaking or rheumatic-heat internal accumulation or damp-heat resistance complex combined into rheumatic-heat arthralgia syndrome; phlegm and blood stasis blocking collaterals or cold-dampness and phlegm blood stasis or phlegm-dampness blocking collaterals or phlegm-dampness and blood stasis or phlegm-dampness cold coagulation or dampness evil blocking or phlegm-damp coagulation combined into phlegm and blood stasis syndrome; deficiency of the liver and kidney, stagnation of tendons and veins, or combined with deficiency of the kidney and blood stasis becomes syndrome of deficiency of the liver and kidney and stasis of tendons and veins [17].

Knee osteoarthritis has a long course of disease, and its pathogenesis is complex, often a combination of multiple diseases. Its dialectical classification is mainly divided into four types: damp-heat obstruction syndrome, blood stasis obstruction syndrome, liver-kidney yin deficiency syndrome, and wind-cold dampness syndrome. From a database of 1270 valid literatures, 100 patients were extracted for analysis. The dialectical analysis is shown in Table 2.

Through descriptive frequency and frequency analysis of the results of DM in Table 2 above, and combined with relevant professional knowledge, this topic further summarizes the results of the ten common clinical syndrome types in this study, and a single syndrome type can be obtained. The frequencies are listed in Table 3 from high to low.

#### 3.4.4. Frequency of Symptoms

This is the frequency table of symptoms and signs of the top 10 patients, as shown in Table 4.

#### 3.4.5. Analysis of Drug Composition

A total of 129 traditional Chinese medicines were involved in the cases that met the inclusion criteria. It is divided into four qi, five flavors, meridian, and medicine. The treatment of knee osteoarthritis is mainly based on warm medicine, followed by the medicine of calm, cool, cold, and heat. Four qi generally means that the medicine usually contains four different medicinal properties; five flavors refer to the medicine containing five different medicinal flavors. Their frequency of use is shown in Figure 4 [18].

#### 3.4.6. Quantitative analysis of Single Drug

Angelica sinensis is an essential medicine for promoting blood circulation, which can be used in the treatment of other medicines for promoting blood circulation and wound healing. To study the effect of Angelica sinensis injection—Achyranthes saponin group and ibuprofen group on rabbit knee arthritis, it is shown that it can effectively reduce the pathological process of chondrocyte apoptosis and improve the pathology of osteoarthritis to a certain extent. In the clinical application of orthopedics, licorice mostly plays the role of reconciling medicinal properties. Its taste is sweet, and qi is harmonious, which can reconcile the medicinal taste and relieve medicinal properties. In the clinical use of drugs with strong medicinal power or biased medicinal properties, compatibility with licorice can play a role in reconciling and relieving.

The decoction or extract of Duhuo has sedative, analgesic, and hypnotic effects. Chuanxiong is known as the “qi medicine in blood” and “hemostatic medicine in gas,” which has the power of regulating blood and ventilation. It is a commonly used medicine in orthopaedics for all kinds of acute and chronic injuries and diseases with stagnant blood stasis and poor qi. The active ingredient of ligustrazine can promote the secretion of anabolic factors in chondrocytes, stimulating cell proliferation, and protein synthesis. Its comparison chart is shown in Figure 5.

Total glucosides of paeony can effectively help improve the condition of patients with osteoarthritis and reduce serum levels. Eucommia ulmoides strengthens tendons and bones, dehumidifies, and relieves pain. It is a good medicine for treating kidney deficiency and weak waist and knee pain. Rehmannia glutinosa is sweet, slightly warm, and returns to the liver and kidney meridians, suggesting that Rehmannia glutinosa has a two-way regulating blood-replenishing effect. Poria is sweet, mild in taste, and flat in nature, and it is widely used in various clinical diseases and is a good product for invigorating the spleen, inducing dampness, and diverting water. Its comparison chart is shown in Figure 6.

#### 3.4.7. Medication Rule Analysis Based on Association Rules and Prescription Rule Based on Association Rule Analysis

The association rule algorithm is a rule-based machine learning algorithm that is able to discover interesting relationships from a large number of databases. The purpose is to identify the rules appearing in the database by using certain metrics, which belongs to the unsupervised machine learning method. The number of support degrees was set to 60 (the support degree was 40.3%), the confidence level was set to 0.90, and the formula of 149 prescriptions was summarized. There are 8 pairs of drugs in total, including 6 drugs [19]. The specific drug combination is shown in Table 5.

“Rule Analysis” is based on “Association Rules.” Figure 7 is a comparison chart of the analysis results of association rules with different support degrees (the support degree in the left picture is 32.6%, and the support degree in the right picture is 47.4%).

#### 3.4.8. Analysis of the Law of Formula Composition Based on Entropy Method

*(1) Interdrug Correlation Analysis Based on Improved Mutual Information Method*. Entropy is a measure of uncertainty. The greater the amount of information, the smaller the uncertainty, and the smaller the entropy; the smaller the amount of information, the greater the uncertainty, and the greater the entropy. After setting the correlation and penalty, start clustering analysis. Afterwards, the correlation between these drugs can be obtained, and the top five drugs are shown in Table 6.

Using the complex system entropy clustering method, some core combinations of drugs can be obtained and displayed in a network, as shown in Figure 8.

*(2) New Square Analysis Based on Unsupervised Entropy Hierarchical Clustering*. Through the unsupervised entropy hierarchical clustering analysis method, on the basis of the core combination, the new combination is further excavated, as shown in Figure 9.

### 3.5. Results

TCM clinical syndrome types are the internal basis of diseases, are the pathological generalizations of pathogenic factors, pathological properties, lesion locations, and pathological trends at a certain stage in the development of the disease, and are the theoretical basis for dialectical treatment. Clinically, only by determining the type of TCM syndromes can we apply syndrome differentiation and treatment. However, it is difficult to unify the standard of syndrome types in clinical practice; so, it is essential to study the types of TCM syndromes in an objective, standardized, and normalized manner. DM technology has improved its research efficiency by 38%.

According to the results of this DM, the statistical analysis points out that most of the patients are compound syndromes with a mixture of deficiency and reality, and the frequency of a single syndrome is lower than that of the compound type. It can be seen that the proportion of liver-kidney deficiency syndrome combined with a single syndrome type accounts for the largest proportion; most of the single syndrome types can be combined with liver-kidney deficiency syndrome. A review of relevant textbooks, literatures, and diagnostic criteria for clinical syndrome types of knee osteoarthritis found that most of them were of a single syndrome type. Combined with the etiology, pathogenesis, epidemiological characteristics of knee osteoarthritis, and the statistical results of this study, it is shown that most of the complex syndrome types are the main types, which is consistent with the actual syndrome types of clinical syndrome differentiation. Through the results of DM and statistical analysis, it is further concluded that the syndrome types have liver and kidney deficiency syndrome, which is consistent with the actual situation of clinical syndrome differentiation and treatment. Therefore, it is of important and far-reaching significance to guide clinical practice and improve the clinical theory level and clinical efficacy. Therefore, it is of great and far-reaching significance to have a relatively standard and standardized research result of this complex syndrome type to guide clinical practice and improve the theoretical level of syndrome and clinical efficacy.

## 4. Conclusions

DM technology has become an important part of TCM modernization technology innovation in the past decade, which will play a great role in promoting the progress of TCM modernization research and the improvement of academic level. The research shows that DM technology is the core of knowledge discovery and is a process of extracting valuable knowledge from the data.

This article is the application of DM technology in the past decade about the prevention of knee osteoarthritis, clinical literature sorting, induction, and analysis. Using the treatment principles of classification results and weights, the classification results of clinical syndrome types and the weights of each syndrome type are inferred according to the frequency of occurrence. However, because the sample number did not meet the ideal requirements, sample randomness is not enough and limited by time and funds; so, no big data collection and sorting. Through DM technology to summarize the experience of famous old Chinese medicine, it can finally be established for an objective, standard, and standard clinical syndrome system. This research result is consistent with clinical syndrome differentiation and treatment and can guide clinical application. However, the experimental samples prepared in the experimental process of this paper are not large enough, and the data processing and classification are not very accurate. Therefore, in the subsequent research, we will go deep into the experimental design part. At the same time, the database further expands the database capacity and improves the physical and chemical examination of patients, and the analysis results will be more scientific and credible.

## Figures and Tables

**Figure 1:** Schematic diagram of removing noisy text from training set during clustering.

**Figure 2:** Sigmoid function graph.

**Figure 3:** Wiring diagram.

**Figure 4:** Distribution frequency map of four qi and five flavors of drugs.

**Figure 5:** Comparison of the dosage of Danggui Duhuo.

**Figure 6:** Comparison of dosage of white peony and tuckahoe.

**Figure 7:** Comparison of different support levels.

**Figure 8:** Core portfolio.

**Figure 9:** New party combination.

**Table 1:** Relationship between patient age and knee osteoarthritis.

Average age	Frequency	Percentage
30-44	28	2.28%
45-60	782	61.57%
Over 60	460	36.15%

**Table 2:** Frequency table of TCM syndrome types.

Syndromes	Frequency	Frequency (%)
Damp-heat paralysis syndrome	32	32%
Liver and kidney deficiency syndrome	28	28%
Wind-cold dampness syndrome	26	26%
Blood stasis syndrome	14	14%

**Table 3:** Frequency of compound syndrome types.

Syndromes	Frequency	Percentage (%)
Liver and kidney deficiency syndrome and muscle and vessel stasis syndrome	385	44.77%
Liver-kidney deficiency syndrome and wind-cold-dampness obstruction syndrome	258	30%
Liver and kidney deficiency syndrome combined with phlegm and blood stasis syndrome	115	13.37%
Liver and kidney deficiency syndrome and qi stagnation and blood stasis syndrome	102	11.86%

**Table 4:** Symptom frequency table.

Syndromes	Frequency	Frequency (%)	Syndromes	Frequency	Frequency (%)
Joint pain	123	94.6	Unfavorable flexion and extension	90	69.2
Aggravation after activity	103	79.2	Rainy days are more serious	82	63.0
Morning stiffness	103	79.2	Swollen joints	49	37.6
Bone rubbing	100	76.9	Limbs are heavy	46	35.3
Joint tenderness	98	75.3	Dry throat	40	30.7

**Table 5:** Analysis of medication patterns (frequency ≥ 60).

Drug pattern	Frequency
Bull knee, Angelica	90
Bull knee, coix seed	78
Angelica, coix seed	75
Bull knee, licorice	72
Angelica, licorice	70
Coix seed, licorice	66
Bull knee, pawpaw	63
Bull knee, Tung leather	60

**Table 6:** Interdrug correlation analysis.

Drug 1	Drug 2	Correlation coefficient
Vaccariae Semen	Chuanxiong Rhizoma	0.1665
Vaccariae Semen	Coix seed	0.1618
Pawpaw	Coix seed	0.1168
Vaccariae Semen	Astragalus	0.1143
Tuckahoe	Astragalus	0.1045

## Data Availability

The data underlying the results presented in the study are available within the manuscript.
